# Cloud Computing into Respiratory Rehabilitation Training-Assisted Treatment of Patients with Pneumonia

This article has been retracted.

**DOI:** 10.1155/2021/5884174

**Published:** 2021-09-27

**Authors:** Yan Yu

**Affiliations:** Thoracic and Cardiac Surgery, Zhujiang Hospital of Southern Medical University, Guangzhou 510000, Guangdong, China

## Abstract

In order to study the therapeutic effect of respiratory rehabilitation training on patients with pneumonia, this paper proposes an integrated adjuvant therapy program based on the cloud computing model. A total of 60 pneumonia patients admitted to Zhujiang Hospital of Southern Medical University from January to July 2020 were selected as the research objects and Southern Medical University pneumonia patients as the research object, to be evenly divided into two groups, each group of 30 people. The control group was treated with conventional anti-infection treatment, and the observation group was treated with supplementary respiratory rehabilitation training on the basis of conventional treatment. The therapeutic effects of the two groups were compared. The results showed that the absorption time of lung lesions was (9.17 ± 3.46) days in the observation group and (13.97 ± 3.07) days in the control group, and the difference between the two groups was statistically significant (*t* = 5.683, *P* < 0.001). Respiratory therapy based on the cloud computing model has the characteristics of integration and extensibility, which can be effectively applied to the treatment effect analysis of patients with pneumonia and is of great significance for the effective analysis of patients' blood gas indexes and lung function indexes.

## 1. Introduction

Pneumonia is an inflammation of the final airway, alveolar, and pulmonary amphids caused by various pathogens, physicochemical factors, immune injuries, allergies, and drugs and is the most common respiratory infectious disease, in the world. There is a high incidence and mortality in the range. With the wide application of mechanical ventilation, ventilator-associated pneumonia, VAPs have become the most common hospital-acquired infection. VAP refers to pneumonia that occurs after the establishment of artificial airway treatment of 48 hours after receiving mechanical ventilation, including pneumonia that occurred within 48 hours of the tube. At present, the incidence of VAP is high, and it is reported that 5%–15% of mechanical ventilation patients occurring abroad may have a VAP, and the mortality rate is about 10%; while the incidence of VAP is 7%. ∼55.8%, the mortality is 9.4%∼51.6%, especially in intensive care unit patients, ICU patients, and severe patients; low-resistance ventilation can directly prolong the mechanical ventilation time of patients by 5.4∼14.5 d, ICU patients by 6.1∼17.6  d, and other wards by 11∼12.5 d, thereby increasing patient hospitalization costs. Therefore, effectively preventing VAP is the focus of intensive care attention.

Since 2008, VAP-related preventive measures have been continuously developed and improved. The 2014 US Health Health Epidemiological Society and the American Infectious Disease Association (AHEA/IDSA) have updated 2008 VAP prevention strategies, including the confirmed prevention of VAP measures, to shorten the adult patient, reduce the hustle care room time, reduce the mortality, and save treatment. Some evidence is less than possible to reduce the incidence of VAP and reduce the residence time and mortality rate of intensive care chamber because of the lack of basic constraints. In Miia Jansson et al.'s cognitive survey of the nurse VAP guide for the intensive care room, the average score rate of the knowledge test is 59.9%. Regarding the guidelines, in the research, the medical staff's unknown rate was as high as 54.5%. Berenholtz's survey report shows that the contents of VAP pilot precautions include as high as 80% of the nursing staff. In China, a study shows that doctors and nurses do not know up to 72.1% and 90.6%, respectively. Low clinical implementation: although the guidelines will bring huge benefits to both doctors and patients, the implementation of the guidelines is not optimistic in clinical practice, as well as the implementation of the intensive guardian guide. European and American experts scholars have attracted attention since the 1990s [1].

## 2. Literature Review

Pulmonary disease is a chronic disease, and patients with pulmonary disease are typical clinical manifestations of the activity of active breathing and sexual weight. Air promotion is the most common first symptom. Hormones and other drugs improve the patient's lung function during the treatment, alleviate the degree of breathing difficulties in patients to alleviate the condition, but when the condition arrives at certain stability, continuing to use hormones and other drugs, the patient's condition will not have obvious improvement, so nondrug methods can improve the symptoms of respiratory difficulties in patients and improve the study of patient life quality. The respiratory function has the contraction strength of the respiratory muscle, eliminating the ineffective effect of the auxiliary respiratory muscle, reducing the oxygen consumption of the respiratory muscle, and increasing the clearance of the airway secretion and the airway defense ability, which can improve the ventilation and ventilation function of the lungs.

The effect of respiratory exercise applied to patients with chronic obstructive pulmonary disease is confirmed by many studies, and there is a role in patients with effective interventions for patients. The research on respiratory function exercise on patients with pulmonary disease is mostly for dustpic lung patients. Ezhov believed that there are important means and measures in the treatment of respiratory function. It is the physiological role and good clinical effect that it produces [2]. Abdominal breathing with diaphragm activity is deep and slow, which can improve the unreasonable shallow breathing method of auxiliary ventilator, while increasing the tidal volume, reducing the invalid dead chamber, increasing the amount of alveolar ventilation. Improving gas distribution, while reducing nonelasticisms to overcome when inhalation, the total power reduction of oxygen consumption and power consumption can make the sputum symptoms alleviate. Tang Jun guided the dust lung patient for functional exercise (abdominal breathing) month, and the results show that the patient's conscious chest tightness, shortness of breath, difficulty breathing, and so forth; the lung ventilation; and ventilation function have been improved. Tsyganova et al. showed that breathing exercise can effectively improve the quality of life of patients with dustpiculmonary [3]. Fang, for the first-month respiratory function exercise for patients with case-free pulmonary fibrosis, compared the clinical symptoms, quality of life, and blood gas analysis before and after exercise, and the results show that the above indicators have improved, so they think that breathing function is special. Patients with sex pulmonary fibrosis have positive significance [4]. Some foreign scholars, such as PT and A, combined with the results of data analysis, found that doctors should strictly control the indications of tracheotomy and prematurely choose tracheotomy to aggravate patients with VAP [5]. The views of Matthias D. are opposite to it. It is believed that the MV patients have continuously used ventilators after the tracheal cut, and the patient's ventilation time has no effect on the occurrence of VAP [6]. Anai et al. showed that the ventilator treatment after tracheal cutting did not only increase the probability of VAP in patients but also exacerbate the patient's condition, and it would like to cause the patient to die [7]. Aoyama et al., with tracheal intubation, showed the initial use of washthaki to clean the oral cavity, which can effectively prevent the occurrence of VAP caused by bacterial oral inflammation. Evidence-based nursing demonstrates that oral care of MV patients can minimize 50% of the VAP incidence, and some scholars have found that high-quality oral care can effectively reduce oral bacteria breeding, and one-third of MV patients can be free from a VAP occurring [8]. Bendib *i* recommended, in terms of oral care frequencies, that MV patients who have VAP should ensure oral care twice a day [9]. In addition, scholars have found that critically ill patients that are using mechanical ventilation treatment are permitted by the patient's condition, with ensuring that patients are often in semisuction positions and can effectively prevent VAP. Zhu et al. found that the biopsy airway is more secure than the physiological saline method in the moisture airway method and can effectively prevent VAP [10]. There is a literature report that the nurse frequent replacement with the disinfection ventilator does not reduce the probability of VAP in patients. Chen et al. stated that nurses should clarify the prevention and nursing measures of VAP, which is of great significance in preventing VAP work. Hospital medical staff should update their VAP-related knowledge regularly. Only when medical staff skillfully master the knowledge and skills of VAP prevention, patients can be better prevented from VAP. The respiratory function, as a pulmonary rehabilitation method, can reduce the clinical symptoms of respiratory diseases, and it is easy to learn, with no creative pain, economically practical, and very good promotion, so this study is to take breathing function exercise rehabilitation effect of patients with interstitial pulmonary diseases to evaluate the effectiveness of respiratory training interventions.

## 3. Data and Methods

### 3.1. General Information

Choosing 60 patients with pneumonia in the Pearl River Hospital of South Medical University from January to July 2020, using a random number of respiratory rehabilitation training groups (observation group, *n* = 30) and conventional respiratory rehabilitation group (control group, *n* = 30). Through cloud computing mode, the respiratory frequency, blood oxygen saturation, Murray lung injury score, Apachei score, and Barthel daily life function were compared (*P* > 0.05). See Table 1.

### 3.2. Incorporation and Exclusion Standard

Inclusion criteria: ①according to the new coronavirus infected pneumonia diagnosis and treatment plan (Trial Sixth Edition) diagnosed as NCP; ②primary school and above; ③18 years old ≤ aged ≤ 85 years old, ④vital signs stable, restless oxygen saturation > 90%; and ⑤ Barthel daily life function rating > 60 by 60. Exclusion criteria: ①severe nervous system lectures; ②mental abnormalities; ③very poor compliance; and ④listening or language dysfunction. All patients need respiratory rehabilitation training based on the guiding principles of sensory tolerance and no decrease in blood oxygen saturation.

### 3.3. Method

Both patients received drug treatment for medical treatment programs issued by NCP Sixth Edition Guidelines for the Office of the National Health and Health Committee Office/National Traditional Chinese Medicine Office Guanda.com [2020] No. 145.

#### 3.3.1. Control Group

On the basis of drug comprehensive treatment, training for patients with traditional respiratory rehabilitation is implemented. Respiratory rehabilitation contents are based on 2019NCP Respiratory Rehabilitation (first edition), combined with internal medicine nursing (sixth edition) including respiratory model training and respiratory rehabilitation. Respiratory mode training includes shrinking breathing, abdominal breathing, and starting training on the second day of the hospital, 3 to 4 times a day, 10∼15 min each time. Respiratory rehabilitation: patients carry out their own positions, sitting and standing positions, split, squats, and raising their legs according to their own conditions, 3 times a day, 5 to 10 min each time. Responsible nurses check the medical respiratory rehabilitation training implementation 2 times a day and fill in the patient's respiratory rehabilitation training execution list, with intervention time 10∼26 d, average (19.00 ± 2.63) *d*.

#### 3.3.2. Observation Group

On the basis of drug comprehensive treatment, patients in the observation group implemented the guidance of breathing rehabilitation training.

(1) Refinement of mission: ①Making a video. In this nursing team, two respiratory nurses are involved, one to demonstrate, one to talk, and then add subtitles and relaxed music to the video; ②establishing an empowering respiratory rehabilitation training patient group, through WeChat push-to-record related videos and urging patients to carry out rehabilitation training every day; ③making color page diagrams, pasting in the eye-catching place of the ward, facilitating patients to watch the imitation exercises at any time.

(2) Implementation of respiratory rehabilitation training: employment rehabilitation respiratory rehabilitation training is implemented on the basis of traditional respiratory rehabilitation by empowering the potential of NCP patients and promoting patient proactive participation in respiratory rehabilitation training and it is actively completed. Specific steps: ①perfect psychological assessment within the 24 hours after admission, understanding the patient's psychological, daily life ability, and cultural level. Positive energy of NCP-related knowledge helps patients establish confidence in victory disease. ② Responsible nurses explain the specific method steps and significance of respiratory rehabilitation training for patients in charge and guide patients to watch the rehabilitation training video pushed by the patient group, make in-depth communication, understand the patient's attitude and will, and actively guide and encourage patients to participate. ③Ending process is a step-by-step process. After the end of the first 2 steps, according to the previous assessment information, they assist patients to develop the target of individual respiratory and the specific implementation plan. This is an important step in the process of communication. In this process, responsible nurses only need to provide technical guidance and theoretical support, with patient's willingness and goals, and formulate practical training programs to make patients actively conduct respiratory rehabilitation training. ④ They evaluate the patient's rehabilitation process, and patients complete a phase goal, moderate praise, and encouragement. In the process of empowering health education, the responsible nurse participates and fills in the plan schedule and respiratory rehabilitation training execution order, with intervention time 7∼21 D, average (16.00 ± 3.24) *d*.

### 3.4. Observation Indicators

Observe the comparison of the two groups of patients during intervention (when admission) and after intervention (1 day before discharge), the dynamic results of Barthel daily life functions, and respiratory rehabilitation training.

### 3.5. Statistical Method

The data are statistically analyzed by SPSS 20.0 software. The measurement data are indicated in $\bar{x}\pm s$, and the two sets of square numbers are compared to the *t*-test; counting data are expressed in a ratio, using the X2 test, which has statistically significant differences in *P* < 0.05.

## 4. Results

### 4.1. Comparison of Observation Indicators before and after Intervention in Two Groups

The two groups of patients were intervened with the respiratory rate and blood oxygen saturation; Barthel scores were compared; and there was no statistical significance (*P* > 0.05). The respiratory frequency, blood oxygen saturation, and Barthel scores were higher than those of the control group, and the difference was statistically significant (*P* < 0.05). The difference between the respiratory frequency, blood oxygen saturation, and Barthel score before and after intervention was statistically significant (*P* < 0.05); see Tables 2–4.

### 4.2. Comparison of Respiratory Rehabilitation Training Compliance in Two Groups

The respiratory rehabilitation training compliance (93.33%) of the observation group was higher than the control group (63.33%), and the difference was statistically significant (*x*^2^ = 7.954, *P*=0.005). See Table 5.

### 4.3. Two Groups of Patients CT Showed Comparison of Pulmonary Lesion Absorption Time

The pulmonary CT in the observation group showed that the absorption time of the pulmonary lesion was (9.17 ± 3.07) *d*, the control group was (13.97 ± 3.07) *d*, and the difference in the two groups was statistically significant (*T* = 5.683, *P* < 0.0011).

## 5. Discussion

Cloud computing's discovery of hidden and neglected related information in a large number of data is of great significance for the early detection and prevention of disease changes and influencing factors in pneumonia patients. After deploying a hospital information system through the cloud computing mode, it is statistics from the system to patients with pneumonia, cough, and chest tightness ratio is higher than ordinary patients, so how to effectively reduce the lung function injury of serious patients, promote early comprehensive rehabilitation of patients, reduce the mortality is the focus difficulty. Respiratory rehabilitation training has the characteristics of target, effectiveness, and the training of patients and patient's physical and mental state can effectively improve lung function and clinical symptoms in patients with infective pneumonia. Employing the concept of health education is to provide patients with the necessary skills, opportunities, and power. With the decent advantage of “power” “ability,” enhancing patient self-care ability and improving the awareness of the disease, this cognitive effect is better than conventional health education, making patients have more waken understanding of disease-related self-behavior improvement, effectively promoting postoperative rehabilitation training in daily behavior, thereby improving the effectiveness of nursing staff to implement the nursing intervention.

Pulmonary disease is a chronic disease. Patients with lung disease have typical clinical manifestations of active dyspnea and progressive aggravation, and the promotion of qi is the most common first symptom. Cloud computing studies show that communication breathing is conducive to improving the self-efficacy of patients with chronic obstructive pulmonary diseases, thereby improving the treatment effect. The results of this study showed that after the observation group was implemented, the respiratory rate, blood oxygen saturation, and Barthel scores were significantly improved, and the difference was statistically significant (*P* < 0.05). The lung inflammatory absorption time of the observation group was shortened, and the difference was statistically significant compared to the control group (*P* < 0.05). In routine nursing, patients' compliance with respiratory rehabilitation training is poor, which may be because NCP is a new and highly infectious disease. Most patients lack medical knowledge and lack confidence in rehabilitation training because they have negative and fear psychology. Studies have shown that empowering education can significantly reduce the psychological state of depression anxiety in patients with polycystic ovary syndrome, improve the patient's self-care ability, and improve the compliance of patients with medical care. This study is the first attempt to apply the communication theory to NCP patient respiratory rehabilitation training. It has a planned guidance for patients to improve self-learning cognition and ability and encourage patients to actively participate in the development of their personal goals and positive feedback encouragement. It fully mobilizes the patient's self-efficacy, and the respiratory rehabilitation training will be passively active, to facilitate the improvement of respiratory rehabilitation training. The results of this study show that the compliance of respiratory rehabilitation training in the observation group is higher than that of the control group, indicating that the respiratory rehabilitation training increases the subjective initiative of NCP patient respiratory rehabilitation training, better compliance with rehabilitation training programs, thus better improving breathing. Respiratory function and quality of daily life have been improved with remarkable results.

## 6. Conclusion

Studies have shown that enabling breathing training is conducive to improving self-efficacy in patients with COPD, thus improving the treatment results. The results showed that after enabling respiratory rehabilitation training, the respiratory frequency, blood oxygen saturation, and Barthel scores were significantly improved compared with the control group (*P* < 0.05). The difference was statistically significant (*P* < 0.05). In summary, through cloud computing, the interior of the hospital and timely data update can be realized, on the one hand, to effectively supervise the treatment of pneumonia in the hospital and, on the other hand, for the application of respiratory rehabilitation training in patients with respiratory failure. In the absence of the patient, the patient's blood gas analysis indicators and lung function can be improved, thereby improving the treatment efficiency.

## Figures and Tables

**Table 1:** Comparison of general information in two groups.

Indicators	Observation group (*n* = 30)	Control group (*n* = 30)
Age (years)	59.00 ± 13.02	56.28 ± 13.75
Respiratory rate (per minute)	24.13 ± 0.78	23.97 ± 0.89
Blood oxygen saturation (%)	92.93 ± 0.98	93.50 ± 0.94
Murray lung injury score (score)	1.40 ± 0.62	1.37 ± 0.56
Apache score II (score)	6.63 ± 0.93	6.53 ± 0.86
Barthel score (score)	79.00 ± 6.49	79.33 ± 4.87

**Table 2:** Comparison of respiratory rate between the two groups before and after intervention ($\bar{x}\pm s$).

Group	Number of cases	Respiratory frequency (times per minute)		
		Before the intervention	After the intervention	Difference
Observation group	30	24.13 ± 0.78	21.90 ± 0.71^*∗*^	2.23 ± 1.07
Control group	30	23.96 ± 0.89	22.47 ± 0.68^*∗*^	1.50 ± 1.04
T value		0.77	3.14	2.68
*P* value		0.44	≤0.01	≤0.01

*Note.*^*∗*^*P* < 0.05 compared with preintervention within the group.

**Table 3:** Comparison of blood oxygen saturation before and after intervention between the two groups ($\bar{x}\pm s$).

Group	Number of cases	Blood oxygen saturation (%)		
		Before the intervention	After the intervention	Difference
Observation group	30	92.93 ± 0.98	97.53 ± 1.50^*∗*^	4.60 ± 1.59
Control group	30	93.03 ± 0.89	94.06 ± 0.87^*∗*^	1.03 ± 1.25
T value		−0.41	10.94	9.67
*P* value		0.68	≤0.001	≤0.001

*Note.*^*∗*^*P* < 0.05 compared with preintervention within the group.

**Table 4:** Comparison of the Barthel scores between the two groups before and after intervention ($\bar{x}\pm s$).

Group	Number of cases	Barthel score (score)		
		Before the intervention	After the intervention	Difference
Observation group	30	79.00 ± 6.49	96.50 ± 3.75^*∗*^	17.50 ± 5.69
Control group	30	79.33 ± 4.86	85.33 ± 4.53^*∗*^	6.00 ± 4.43
T value		−0.22	10.39	−8.73
*P* value		0.82	≤0.001	≤0.001

*Note.*^*∗*^*P* < 0.05 compared with preintervention within the group.

**Table 5:** Comparison of respiratory rehabilitation training compliance in two groups (example (%)).

Group	Observation group	Control group
Number of cases	30	30
Compliance	28 (93.33)	19 (63.33)
Nonadherence	2 (6.67)	11 (36.67)

## Data Availability

The data used to support the findings of this study are available from the corresponding author upon request.
